This article has been retracted.

# Functional screen analysis reveals miR-3142 as central regulator in chemoresistance and proliferation through activation of the PTEN-AKT pathway in CML

**DOI:** 10.1038/cddis.2017.223

**Published:** 2017-05-25

**Authors:** Lifen Zhao, Yujia Shan, Bing Liu, Yang Li, Li Jia

**Affiliations:** 1 College of Laboratory Medicine, Dalian Medical University, Dalian 116044, Liaoning Province, China

## Abstract

Chronic myeloid leukemia (CML) is caused by the constitutively active BCR-ABL tyrosine kinase. Although great progress has been made for improvement in clinical treatment during the past decades, it is common for patients to develop chemotherapy resistance. Therefore, further exploring novel therapeutic strategies are still crucial for improving disease outcome. MicroRNAs (miRNAs) represent a novel class of genes that function as negative regulators of gene expression. Recently, miRNAs have been implicated in several cancers. Previously, we identified 41 miRNAs that were dysregulated in resistant compared with adriamycin (ADR)-sensitive parental cells in CML. In the present study, we reported that miR-3142 are overexpressed in ADR-resistant K562/ADR cells and CML/multiple drug resistance patients, as compared with K562 cells and CML patients. Upregulation of miR-3142 in K562 cells accelerated colony formation ability and enhanced resisitance to ADR *in vitro*. Conversely, inhibition of miR-3142 expression in K562/ADR cells decreased colony-formation ability and enhanced sensitivity to ADR *in vitro* and *in vivo*. Significantly, our results showed miR-3142-induced ADR resistance through targeting phosphatase and tensin homologue deleted on chromosome 10 (PTEN), which led to downregulation of PTEN protein and activation of PI3 kinase (PI3K)/Akt pathway. Inhibition of Akt using Akt inhibitor or introduction of PTEN largely abrogated miR-3142-induced resistance. These findings indicated that miR-3142 induces cell proliferation and ADR resistance primarily through targeting the PTEN/PI3K/Akt pathway and implicate the potential application of miR-3142 in cancer therapy.

Chronic myeloid leukemia (CML) is a malignant disease of a primitive hematopoietic cell, characterized by a reciprocal translocation between chromosomes 9 and 22, and creates the fusion gene *BCR-ABL1*, which is a deregulated tyrosine kinase that drives the leukemia.^1^ CML treatment has been significantly improved. However, a significant percentage of the patients with CML failed to respond effectively to the current regimen of drug therapy including frontline tyrosine kinase inhibitors (TKIs) therapy and had to be considered for allogeneic stem cell transplantation, which has a high risk of morbidity and mortality.^2, 3, 4^ MDR1 encodes a 170 kDa transmembrane protein, P-glycoprotein (P-gp), which causes the efflux of antineoplastic agents from tumor cells via an adenosine triphosphate-dependent process. Overexpression of P-gp protein is one of the major mechanisms for multiple drug resistance (MDR) in cancer cells. The question of whether P-gp could mediate resistance to imatinib was clinically important and have been elucidated.^5^Moreover, multifactorial causes for inadequate response to imatinib and nilotinib are discussed: acquired somatic mutations in the BCR-ABL kinase domain impairing drug binding are the most common^6, 7^ among others, such as BCR-ABL overexpression,^8^ centrosomal aberrations,^9^ clonal evolution^10, 11^ and the bypass of BCR-ABL signaling pathways.^12^ Recently, it was reported that type of BCR-ABL transcript may impact the probability of response to TKI among patients with CML treated with various TKI regimens.^13^ Therefore, it is critical to continue research into novel therapeutic approaches.

MicroRNAs (miRNAs) are endogenous, ~22-nucleotide-length small RNA molecules that negatively regulate the gene expression by directly targeting the 3′- untranslated region (3′-UTR) of mRNAs.^14^ MiRNAs regulate the expression of a wide variety of target genes and aberrant expression of miRNAs functions as tumor suppressors or oncogenes according to the role of their target genes.^15, 16^ Increasingly, miRNAs are involved in modulating cancer cell behavior, including cell proliferation and apoptosis, cell cycle and differentiation.^17^ Dysregulated miRNA expression is a common feature of solid and hematopoietic malignancies.^18, 19^ Nevertheless, miRNA expression in chemoresistant CML is not widely investigated and the mechanisms that underlie aberrant miRNAs expression are not well understood.

Phosphatase and tensin homologue deleted on chromosome 10 (PTEN) is one of the most commonly altered tumor suppressors in human cancers and a key regulator of cell growth and apoptosis.^20^ Functionally, PTEN converts phosphatidylinositol-3,4,5-trisphosphate in the cytoplasm to phosphatidylinositol-4,5-bisphosphate, thereby directly antagonizing the activity of PI3 kinase (PI3K).^21^ Its inactivation results in constitutive activation of the PI3K/AKT pathway and in subsequent increase in protein synthesis, cell cycle progression, migration and survival.^22^ Recent studies have revealed that miRNAs could mediate the oncogenic function of the Akt pathway in several cellular processes, including cell proliferation, epithelial–mesenchymal transition and tumour angiogenesis, in breast, colon and lung cancers.^23, 24^ However, the function of the miRNA/PTEN/Akt pathway during CML chemosensitivity is poorly investigated.

Here we examined the relationship between miR-3142 and PTEN in CML and found an atypical miR-3142-PTEN-AKT pathway. Inhibition of this pathway suppresses proliferation and sensitizes CML cells to ADR. Altogether, these results provide a mechanism by which miR-3142 modulates CML cell proliferation and chemosensitivity.

## Results

### Differential miR-3142 expression in K562–ADR-sensitive, -resistant CML cells and CML patients

Previously, we identified 41 miRNAs that were dysregulated in resistant compared with adriamycin (ADR)-sensitive parental cells in CML.^25^ Among these candidate miRNAs, miR-3142 were expressed at significantly higher levels in ADR-resistant CML cells. In this study, we assessed the expression levels of miR-3142 using real-time quantitative RT-PCR (qRT-PCR). As expected, miR-3142 was significantly downregulated in K562 and KU812 cells as compared with K562/ADR, KU812/ADR cells (Figure 1a). Then, the expression levels of miR-3142 were analyzed in 36 CML patients. As expected, miR-3142 were significantly downregulated in CML patients compared with that in CML/MDR patients (Figure 1b). These data suggested that alterations of miR-3142 may be involved in the chemoresistance of CML.

### miR-3142 inhibited expression of PTEN and bound to the 3′-UTRs

We next examined its potential targets by searching the TargetScan, PicTar and miRNA.org. Among the search results, we identified *PTEN* as a theoretical target gene of miR-3142. A dual-luciferase reporting system was used to examine whether miR-3142 affected PTEN by directly targeting this specific complementary sequence in its 3′-UTR region. As shown in Figure 2a, miR-3142 transfection imposed a reduction in the luciferase activities. The suppressive effects of miR-3142 on luciferase activities were completely deprived by introduction of nucleotide mutations in PTEN-3′-UTR, suggesting an importance of appropriate binding of miR-3142 to the target 3′-UTRs. The expression level of *PTEN* was detected in CML patients and CML cells by qPCR. As shown in Figures 2b and c, the mRNA level of *PTEN* was higher in CML and K562 cells than in CML/MDR and K562/ADR cells. Moreover, there was a strong negative correlation between Log2-transformed miR-3142 expression and Log2-transformed *PTEN* expression in CML patients (*r*=−0.83, *P*<0.01) (Figure 2d). To validate that *PTEN* was a direct target of miR-3142, we analyzed PTEN expression after miR-3142 or Anti3142 transfection. We found that transfection of miR-3142 reduced, but Anti3142 increased both the protein and mRNA levels of *PTEN* (Figures 2g and h). In addition, the engineered levels of miR-3142 expression in the above transfection with miR-3142 or Anti3142 were confirmed (Figure 2e).

### Ectopic expression of miR-3142 in K562 cells enhanced chemoresistance and stimulated proliferation

We next analyzed the effects of miR-3142 on ADR resistance and cell proliferation. K562 cells were transfected with miR-3142 mimic, negative control (NC), respectively. The upregulation of miR-3142 was confirmed by qRT-PCR (Figure 2e). ADR sensitivity was analyzed by CCK-8 and FACS analysis. Results showed that transfection of miR-3142 in K562 cells could increase cell viability and reduced cell apoptosis (Figures 3a and b). In addition, induction of apoptosis was further assessed by detection of the active form of caspase-3 and poly (ADP-ribose) polymerase (PARP). As shown in Figure 3c, upregulation of miR-3142 led to reduced protein levels of cleaved caspase 3 and PARP. Furthermore, the effect on cell proliferation was further confirmed. The proliferation rate of miR-3142 expressing cells was significantly increased (Figure 3d). According to this, we could show strongly increased colony-forming capacity of K562 cells after overexpression of miR-3142 (Figure 3e).

### Knockdown of miR-3142 in K562/ADR cells inhibited chemoresistance and proliferation

To further investigate the effects of miR-3142 downregulation on the sensitivity and cell proliferation of CML cells, K562/ADR cells were transfected with Anti3142 or control, respectively. The downregulation of miR-3142 was confirmed by qRT-PCR (Figure 2e). As shown in Figure 4a, Anti3142 could reduce the cell vialibity in K562/ADR cells by CCK-8 analysis, in comparison with the control-transfected cells. Moreover, results showed that the rate of apoptosis was significantly higher when miR-3142 was inhibited in K562/ADR cells (Figure 4b). Consistently, induction of cleaved caspase 3 and PARP was significantly increased in miR-3142 downregulation cells as compared with the control cells (Figure 4c). Furthermore, the proliferation rate of miR-3142-expressing cells was significantly reduced (Figure 4d). According to this, we could show strongly reduced colony-forming capacity of K562/ADR cells after knockdown of miR-3142 (Figure 4e).

### PI3K/Akt signaling contributed to miR-3142-mediated chemoresistance and cell proliferation

In addition, the phosphorylation levels of Akt, a major target of PTEN^26^ and a critical molecule in tumor development, cell survival and proliferation,^27^ were elevated by ectopic expression of miR-3142 and decreased by knockdown of miR-3142 (Figure 5a). Moreover, we determined the effect of miR-3142-mediated suppression of PTEN on the downstream pathway genes. Results indicated that decreased p21, p27 and increased cyclin D1 expression could be caused by miR-3142 overexpression in K562 cells, whereas opposite effects on the regulation of p21, p27 and cyclin D1 were found when miR-3142 was knocked down in K562/ADR cells (Figure 5a). Ectopic expression of miR-3142 reduced PTEN expression leading to activation of PI3K/Akt pathway (Figure 5a), promotion of the cell viability, colony-forming ability and inhibition of the ADR-induced cell apoptosis. We next tested the role of PI3K/Akt signaling in regulation chemoresistance and proliferation by miR-3142. miR-3142-transfected K562 cells were treated with Akt shRNA or PI3K inhibitor LY294002. As shown in Figures 5b and c, Akt shRNA/ LY294002 abrogated miR-3142-activated Akt and inhibited miR-3142-induced ADR resistance, as indicated by a decrease in cell viability and an increase in apoptosis. In addition, Akt shRNA/ LY294002 abrogated miR-3142-activated Akt and inhibited miR-3142-induced enhanced cell proliferation, as indicated by a decrease in colony-forming ability and proliferation rate. Furthermore, the protein levels of the main signal molecules of PI3K/Akt pathway were analyzed by western blotting. Our results indicated that in K562-miR-3142 cells, the protein levels of PI3K/Akt pathway were decreased in Akt shRNA/ LY294002 treatment group compared with control group (Figure 5f). These data suggested that miR-3142 promoted chemoresistance and proliferation by simultaneously activating PI3K/Akt pathway.

### Repression of PTEN was essential for miR-205-induced proliferation and chemoresistance

Then, we examined whether repression of PTEN was essential for miR-3142-induced cell survival. Plasmid vectors expressing PTEN were constructed. Ectopic delivery of PTEN inhibited cell proliferation and increased sensitivity to ADR in K562/ADR cells (Figures 6e–h). Moreover, downregulation of PTEN in K562 cells exerted opposite effects (Figures 6a–d). In addition, compared with the control group, reexpression of PTEN could inhibit cell viability and increase apoptosis rates of K562 cells induced by miR-3142 (Figures 6a–d). Conversely, silencing PTEN in Anti3142-transduced cells could promote cell viability and suppress apoptosis rates (Figures 6e–h). More importantly, restoration of PTEN decreased Akt activation induced by miR-3142 (Figure 6i). Conversely, silencing PTEN in K562/ADR-Anti3142 cells exhibited opposite effects (Figure 6j). These data supported that downregulation of PTEN was essential for miR-3142-induced increase of chemoresisitance and proliferation in CML.

### Knockdown of miR-3142 in K562/ADR cells inhibited tumor growth *in vivo*

To confirm the effect of miR-3142 on CML cell chemosensitivity and cell growth *in vivo*, we also performed *in-vivo* experiment. As shown in Figure 7a, tumors grow at a slower rate in Anti3142 cells than control cells. Significantly, the combined Anti3142 and ADR treatment markedly restricted the tumor growth to low volumes. In addition, decreases in weights of tumors excised from animals of the Anti3142 group were also observed as compared with those of the control group (Figure 7b). Consistent with the above observations, tumors injected with Anti3142 had decreased Ki67 (Figure 7c). Moreover, significant higher protein levels of PTEN were shown in Anti3142-transduced tumors (Figure 7c). These results confirmed the *in vitro* tumor suppressive effect of downregulation of miR-3142 in a prostate xenograft model.

## Discussion

In our preliminary screening analysis, we found miR-3142 to be upregulated in K562/ADR cells compared with K562 cells.^27^ In the current study, we confirmed a higher level of miR-3142 expression in K562/ADR cells and CML/MDR patients than that in K562 cell and CML patients. Here we showed a tumor-promoting role of miR-3142 in CML, overexpression of which robustly promotes cell proliferation and enhanced resistance to ADR *in vitro*. In contrast, inhibition of endogenous miR-3142 decreased cell proliferation and enhanced sensitivity to ADR *in vitro* and *in vivo*. At the molecular level, the PI3K/ AKT pathways contribute to miR-3142-mediated resistance of CML cells, likely mediated by suppressing PTEN expression. Of note, the close correlation between high miR-3142 expression and low expression of PTEN were confirmed in CML cells and in CML patient samples.

Resistance to chemotherapy may arise from inherent genetic instability or through selection of environmental stress. Recently, miRNAs have emerged as crucial mediators in regulating the cellular responses of cancer cells to therapy. Patient response to chemotherapy has shown to be closely correlated to the functional status of miRNAs.^28, 29, 30^ It has been reported that miR-214 induces cell survival and chemoresistance.^31^ miRNA-17-5p promoted chemotherapeutic drug resistance of colorectal cancer.^32^ In addition, enforced expression of miR-146a in AML cells lines inhibited cell proliferation and increased sensitivity to antileukemic drugs.^33^ Inhibition of miR-486-5p reduced CML progenitor growth and enhanced apoptosis following imatinib treatment.^34^ miR-30a interfered with the effectiveness of imatinib-mediated apoptosis by an autophagy-dependent pathway in CML.^35^ Enforced expression of miR-424/miR-30e was shown to suppress proliferation and induce apoptosis of K562 cells.^36, 37^

Thus, miRNAs are increasingly viewed as potential diagnostic and therapeutic tools. Our results revealed that miR-3142 expression was significantly upregulated in K562/ADR cells and CML/MDR patients compared with K562 cell and CML patients. In addition, inhibition of endogenous miR-3142 in K562/ADR cells suppressed proliferation and sensitized them to ADR treatment *in vitro*. In contrast, restoration of miR-3142 expression in K562 cells remarkably promoted proliferation and reduced chemosensitivity *in vitro*. Moreover, we demonstrated that downregulation of miR-3142 suppressed cell growth and enhanced chemosensitivity *in vivo.*

*PTEN* acts as a tumor suppressor gene through inhibition of PI3K/AKT, which regulates cellular growth, metabolism and survival. Recent studies have demonstrated the inactivation of PTEN in lung cancer,^38^ breast cancer,^39^ glioblastomas,^40^ endometrial carcinoma,^41^ colorectal carcinoma^42^ and hematologic malignancies.^43, 44^ Inactivation of the tumor suppressor PTEN renders cells vulnerable to malignant transformation; however, additional oncogene activation is frequently necessary to drive forward the transformation process.^45^ miR-19b overexpression reduced H2O2-induced apoptosis and improved cell survival in H9C2 cardiomyocytes by silencing PTEN.^46^ The Mir-17-5p/PTEN axis has been reported to be highly related to chemoresistance in prostate cancer and pancreatic cancer.^47, 48^ Inhibition of miR-26a or miR-214 could induce more apoptosis in primary cultured CLL cells via downregulate expression of PTEN.^49^ In this report, we utilized *in silico* algorithms to find miR-3142 target genes in the PI3K/ Akt survival pathway and found that PTEN was a potential target of miR-3142. Upregulation of *PTEN* mRNA and protein was detected after repression of miR-3142 in K562/ADR cells. In addition, downregulation of *PTEN* mRNA and protein was detected after overexpression of miR-3142 in K562 cells. Luciferase reporter assays confirmed that *PTEN* was a direct target gene of miR-3142. We also found that miR-3142 mediated induction of PTEN, leading to activation of the PI3K/AKT pathway. Our observations also indicated that PTEN overexpression could reverse many of the biological effects of miR-3142. These results indicated that miR-3142 had an important role in ADR resistance by targeting PTEN/PI3K/Akt pathway. It was possible that miR-3142 might also target additional target genes, as a single miRNA can target a broad range of molecular regulators in a context-dependent manner. Thus, further investigations were required.

In summary, this study suggested that miR-3142 was upregulated in K562/ADR cells and CML/MDR patients. Alteration of miR-3142 seemed to be associated with chemoresistance and cell proliferation. We also provided results demonstrating that miR-214 induced cell proliferation and ADR resistance by targeting the PTEN/PI3K/Akt pathway. Therefore, miRNA-3142 could have a potential target for CML therapeutic intervention.

## Materials and methods

### Cell lines and patient samples

CML in blast crisis cell lines K562, KU812 were maintained in a RPMI-1640 medium containing 10% fetal bovine serum (FBS), 100 U/ml penicillin and 100 *μ*g/ml streptomycin at 37 °C in a 5% CO_2_ humidified atmosphere. The ADR-resistant cell lines K562/ADR and KU812/ADR were incubated in the presence of ADR (Sigma, St Louis, MO, USA; 1 *μ*g/ml) until at least 3 days before starting the experiments. A total of 36 CML patients from the First Affiliated Hospital of Dalian Medical University (Dalian, China) were enrolled in the study. The diagnosis of CML was based on cytomorphology, cytochemistry, multiparameter flow cytometry, immunology, molecular genetics and cytogenetics. Written informed consent was obtained from all of the patients and the study were approved by and the institutional human ethical committee. Peripheral blood mononuclear cells (PBMCs) were isolated from patient blood using Ficoll-Hypaque solution according to manufacturer’s instructions (StemCell Technologies, Inc., Vancouver, BC, Canada). The membrane expression of P-gp was studied with flow cytometry. Furthermore, the PBMCs were divided into two groups, CML without MDR (multidrug resistance, *n*=16) and CML/MDR(*n*=20). The clinical data of enrolled 36 patients was given in Supplementary Table 1.

### Real-time PCR assay

Total RNA was extracted using Trizol reagent (Invitrogen, Carlsbad, CA, USA) according to the manufacturer’s instructions. After reverse transcription, the levels of PTEN mRNA were determined using SYBR-Green real-time PCR assay (Takara, Dalian, China). The levels of PTEN mRNA were normalized to that of GAPDH and the fold change was calculated using the 2–ΔΔCT method. For miRNA detection, a miRNA-specific TaqMan MiRNA Assay Kit (Applied Biosystems, Forster, CA, USA) was used according to the manufacturer’s instructions. Endogenous U6 small nuclear RNA was detected as an internal control. The delta Ct values were normalized to those obtained from the amplification of endogenous U6 small nuclear RNA. All of the reactions were performed triplicate.

### Colony assay

This was performed to measure the capacity of cell proliferation. After transfection, the cells (1 × 10^3^) were mixed completely with RPM-1640 medium containing 0.9% methylcellulose solution (MethoCult TM H4100; StemCell Technologies), 10% FBS and seeded onto 24-well plates. Single cells were randomly and evenly distributed throughout the wells. Colonies were formed and counted 1 week later using an inverted microscope (Olympus, Tokyo, Japan). The number of colonies containing more than 50 cells was counted. All analyses were performed in triplicate.

### Western blot assay

The cells were lysed in RIPA buffer with protease and phosphatase inhibitors (Roche, Beijing, China). The protein was separated in a 10% polyacrylamide gel and transferred to a methanol-activated PVDF membrane (Millipore, Beijing, China). The membrane was blocked for 2 h in Tris-buffered saline Tween-20 containing 5% skimmed milk and then probed with caspase-3, cleaved 85 kDa fragment of PARP, PARP, cleaved, active caspase-3 (Cell Signaling Technology, Beverly, MA, USA), anti-Akt, anti-phospho-Akt 308 and anti-phospho-Akt 473 (Abgent, San Diego, USA), anti-p21, anti-p27, anti-cyclinD1 and anti-PTEN (Abcam, Cambridge, UK) and GAPDH (Bioworld, Nanjing, China) overnight at 4 °C. After a 1 h incubation with anti-mouse or anti-rabbit HRP-conjugated secondary antibody, the protein level was detected.

### Apoptosis assay

Cell apoptosis was evaluated using an Annexin-V-FITC apoptosis detection kit (BD, Franklin Lakes, NJ, USA). Briefly, after treatment with chemotherapeutic agents (K562/ADR, ADR-40 *μ*g/ml; K562, ADR-1 *μ*g/ml) for 48 h, cells were collected, resuspended in 100 *μ*l flow cytometry binding buffer and stained with 5 *μ*l Annexin V/FITC followed by 5 *μ*l PI. Cells were then incubated in the dark for 15 min at room temperature and 400 *μ*l binding buffer was added. The cells were immediately measured by FACSCalibur (Becton-Dickinson, Franklin Lakes, NJ, USA).

### Immunohistochemistry

At the end of observation, animals were killed and tumors were retrieved for further analysis. Tumors were immediately immersed in 4% buffered formaldehyde, washed, dehydrated and finally embedded in paraffin. Tumor slices were deparaffinized. After washing steps, peroxidase blocking was carried out for 10 min to quench the endogenous peroxidase. Tumors were again washed and then incubated with the primary antibodies at 4 °C overnight. The secondary streptavidin-horseradish peroxidase-conjugated antibody staining was performed at room temperature, visualized in 3,3′-diaminobenzidine (ZLI9018, ZSGB-BIO, Beijing, China), counterstained with hematoxylin, dehydrated and mounted for visualization.

### Viability assay

The cell viability was monitored using the Cell Counting Kit-8 (CCK8) (Dojindo Molecular Technologies, Kumamoto, Japan) according to the manufacturer’s protocol. Briefly, cells (1 × 104) were plated in 96-well plate. Cells were incubated in the presence of different concentrations of ADR. After 48 h of incubation, 10 *μ*l CCK8 reagent was added to the plate. The spectrometric absorbance was measured at 490 nm by microplate reader (Model 680; Bio-Rad, Hercules, CA, USA). All of the experiments were repeated at least three times.

### Plasmids, oligonucleotides, shRNA and transfection

Sequences used were as follows: miR-3142 mimics (miR-3142): 5′-AAGGCCUUUCUGAACCUUCAGA-3′ NC oligo-nucleotides: 5′-UUCUCCGAACGUGUCACGUTT-3′ Anti3142: 5′-UCUGAAGGUUCAGAAAGGCCUU-3′ NC (Control): 5′-CAGUACUUUUGUGUAGUACAA-3′ PTEN-shRNA: 5′-GGCGUAUACAGGAACAAUATT-3′ and NC-shRNA: 5′-ACTCTATCTGCACGCTGAC-3′. These oligonucleotides, PTEN cDNA expression construct and control were purchased from Guangzhou Ribo BioCoLTD (Guangzhou, China). Transfection was performed using the Lipofectamine 2000 reagent (Invitrogen) according to the manufacturer’s instruction.

### Luciferase assay

A pmirGLO Dual-Luciferase miRNA target Expression Vector was used for 3′ UTR Luciferase assays (Promega, Madison, WI, USA). The plasmid pMIR-REPORT-PTEN wt or pMIR-REPORT-PTEN mut was transfected into HEK-293 cells cells together with miR-3142 mimics or the control. *Renilla* was used as a transfection control. Firefly and *Renilla* luciferase activity was measured 48 h after transfection. Data are presented as the mean value±SD for triplicate experiments.

### Xenograft model in nude mice

Nude mice (4 weeks old) were purchased from the Animal Facility of Dalian Medical University and housed in barrier facilities on a 12 h light/dark cycle. The mice were randomly assigned to groups (*n*=6/group). The mice in groups were inoculated subcutaneously with K562/ADR cells (1 × 10^7^) in the right flank and, 1 week later, injected intratumorally with Anti3142 or control three times per week for 3 weeks, combining with intraperitoneal injection of doxorubicin (7 mg/kg) weekly. Tumors were examined every 6 days. Tumor was weighed and tumor volume was calculated using the equation (length × width^2^)/2.

### Statistical analysis

Data are expressed as mean±SD of ⩾3 separate experiments. SPSS17.0 software (SPSS Inc., Chicago, IL, USA) was used for statistical analysis. Multiple group comparisons were analyzed with one-way ANOVA; two-group comparisons were performed with Student’s *t*-test. Correlations between miRNA expression and TP53 status were assessed using Mann–Whitney non-parametric tests. A *P-*value of 0.05 or less was considered significant (*).

## Figures and Tables

**Figure 1:** Differential miR-3142 expression in K562–ADR-sensitive, -resistant CML cells and CML patients. (**a**) qPCR for miR-3142 in K562, KU812 cells and their ADR-resistant cells. (**b**) qPCR for miR-181a in PBMCs from CML patients. qPCR validation of miR-3142 expression levels significantly higher in ADR-resistant cells and chemoresistant cancer samples. *P<0.05. Results are representative of three experiments

**Figure 2:** PTEN was a target of miR-3142. (**a**) The predicted binding sequence of miR-3142 within human PTEN 3′-UTR. (**b**) Luciferase activity analysis of PTEN 3′-UTR (wild type and mutant constructs) after co-transfection with miR-222 in HEK-293 cells. (**b** and **c**) qPCR for *PTEN* in CML cells and CML patients. (**d**) The association between Log2-transformed miR-3142 expression and Log2-transformed *PTEN* expression in CML patients was calculated statistically by using the Pearson’s correlation coefficient (*r*) and the respective *P*-value. (**e** and **f**) K562 cells were transfected with miR-3142 or NC; K562/ADR cells were transfected with Anti3142 or control. miR-3142 expression level was significantly increased after transfection of miR-3142 in K562 cells as measured by qPCR. miR-3142 expression level was significantly decreased after transfection of Anti3142 in K562/ADR cells. (**g** and **h**) qPCR and western blotting for PTEN expression in indicated cells. Values are shown as mean±SD of three independent experiments. *P<0.05

**Figure 3:** Ectopic expression of miR-3142 in K562 cells enhanced chemoresistance and stimulated proliferation. (**a**) K562 cells transfected with either miR-3142 or NC. Viability was determined with an CCK-8 assay as described in Materials and Methods. Data are shown as mean±SD of values from three independent experiments. *P<0.05. (**b**) Cells were then exposed to indicated doses of ADR. Apoptosis was determined by flow cytometric analysis of Annexin-V/PI staining and (**c**) western blot analysis of caspase-3, cleaved caspase-3, PARP and cleaved-PARP. (**d**) CCK-8 assay reveals cell growth curves. (**e**) Representative micrographs (left) and relative quantification (right) of cell colonies analyzed by colony formation assay. Values are shown as mean±SD of three independent experiments. *P<0.05

**Figure 4:** Knockdown of miR-3142 in K562/ADR cells inhibited chemoresistance and proliferation. (**a**) K562/ADR cells were transfected with either Anti3142 or control. Viability was determined with an CCK-8 assay as described in Materials and Methods. (**b**) Cells were then exposed to indicated doses of ADR. Apoptosis was determined by flow cytometric analysis of Annexin-V/PI staining and (**c**) western blot analysis of caspase-3, cleaved caspase-3, PARP and cleaved-PARP. (**d**) CCK-8 assay reveals cell growth curves. (**e**) Representative micrographs (left) and relative quantification (right) of cell colonies analyzed by colony formation assay. Data are shown as mean±SD of values from three independent experiments. *P<0.05

**Figure 5:** PI3K/Akt signaling contributed to miR-3142-mediated chemoresistance and cell proliferation. (**a** and **f**) miR-3142-transduced cells were pretreated with PI3K inhibitor LY294002 or AKT shRNA. Western blot analysis of PTEN, total AKT, phosphoAKT-308, phosphoAKT-473, CyclinD1, p27 and p21 in indicated cells. Results show three identical experiments (bars: mean±SD; *P<0.05). (**b** and **d**) CCK-8 assay shows cell viability and cell proliferation. (**c**) Apoptosis was determined by flow cytometric analysis of Annexin-V/PI staining. (**e**) Relative quantification of cell colonies analyzed by colony formation assay. Data are shown as mean±SD of values from three independent experiments. *P<0.05

**Figure 6:** Restoration of PTEN inversed miR-3142-induced proliferation and ADR resistance. miR-3142-overexpressing cells were transduced with PTEN or control vector. K562 cells were transfected with PTEN-shRNA or NC-shRNA. miR-205 knockdown cells were transduced with PTEN-shRNA or NC-shRNA. K562/ADR cells were transfected with PTEN. (**a** and **e**)Viability was determined with an CCK-8 assay. (**b** and **f**) Apoptosis was determined by flow cytometric analysis of Annexin-V/PI staining. (**c** and **g**) CCK-8 assay reveals cell growth curves. (**d** and **h**) Relative quantification of cell colonies analyzed by colony formation assay. (**i** and **j**) Western blot analysis of PTEN, total AKT,phosphoAKT-308, phosphoAKT-473, CyclinD1, p27 and p21 in indicated cells

**Figure 7:** Downregulation of miR-3142 in K562/ADR cells inhibited growth and enhanced chemosensitivity *in vivo*. (**a**)Tumor growth curves in mice (*n*=6/group) inoculated with indicated cells at indicated days. (**b**) At the experimental endpoint, tumors were dissected and weighed as indicated. (**c**) Immunohistochemically stained for Ki-67 and PTEN are quantified by staining intensity. (**d**) Expression levels of Ki67and PTEN signaling molecules

## References

[bib1] Ben-Neriah Y, Daley GQ, Mes-Masson AM, Witte ON, Baltimore D. The chronic myelogenous leukemia-specific P210 protein is the product of the bcr/abl hybrid gene. Science 1986; 233: 212–214.346017610.1126/science.3460176

[bib2] Jabbour E, Kantarjian H. Chronic myeloid leukemia: 2014 update on diagnosis, monitoring, and management. Am J Hematol 2014; 89: 547–556.2472919610.1002/ajh.23691

[bib3] Dickinson AM, Pearce KF, Norden J, O'Brien SG, Holler E, Bickeboller H et al. Impact of genomic risk factors on outcome after hematopoietic stem cell transplantation for patients with chronic myeloid leukemia. Haematologica 2010; 95: 922–927.2030514310.3324/haematol.2009.016220PMC2878789

[bib4] Hoglund M, Sandin F, Hellstrom K, Bjoreman M, Bjorkholm M, Brune M et al. Tyrosine kinase inhibitor usage, treatment outcome, and prognostic scores in CML: report from the population-based Swedish CML registry. Blood 2013; 122: 1284–1292.2384349410.1182/blood-2013-04-495598PMC3744993

[bib5] Ferrao PT, Frost MJ, Siah SP, Ashman LK. Overexpression of P-glycoprotein in K562 cells does not confer resistance to the growth inhibitory effects of imatinib (STI571) *in vitro*. Blood 2003; 102: 4499–4503.1288132110.1182/blood-2003-01-0083

[bib6] Gorre ME, Mohammed M, Ellwood K, Hsu N, Paquette R, Rao PN et al. Clinical resistance to STI-571 cancer therapy caused by BCR-ABL gene mutation or amplification. Science (New York, NY) 2001; 293: 876–880.10.1126/science.106253811423618

[bib7] Hochhaus A, La Rosee P. Imatinib therapy in chronic myelogenous leukemia: strategies to avoid and overcome resistance. Leukemia 2004; 18: 1321–1331.1521587610.1038/sj.leu.2403426

[bib8] Mahon FX, Deininger MW, Schultheis B, Chabrol J, Reiffers J, Goldman JM et al. Selection and characterization of BCR-ABL positive cell lines with differential sensitivity to the tyrosine kinase inhibitor STI571: diverse mechanisms of resistance. Blood 2000; 96: 1070–1079.10910924

[bib9] Fabarius A, Giehl M, Frank O, Spiess B, Zheng C, Muller MC et al. Centrosome aberrations after nilotinib and imatinib treatment *in vitro* are associated with mitotic spindle defects and genetic instability. Br J Haematol 2007; 138: 369–373.1761482410.1111/j.1365-2141.2007.06678.x

[bib10] O'Dwyer ME, Mauro MJ, Kurilik G, Mori M, Balleisen S, Olson S et al. The impact of clonal evolution on response to imatinib mesylate (STI571) in accelerated phase CML. Blood 2002; 100: 1628–1633.1217688110.1182/blood-2002-03-0777

[bib11] Lahaye T, Riehm B, Berger U, Paschka P, Muller MC, Kreil S et al. Response and resistance in 300 patients with BCR-ABL-positive leukemias treated with imatinib in a single center: a 4.5-year follow-up. Cancer 2005; 103: 1659–1669.1574737610.1002/cncr.20922

[bib12] Mahon FX, Hayette S, Lagarde V, Belloc F, Turcq B, Nicolini F et al. Evidence that resistance to nilotinib may be due to BCR-ABL, Pgp, or Src kinase overexpression. Cancer Res 2008; 68: 9809–9816.1904716010.1158/0008-5472.CAN-08-1008

[bib13] Jain P, Kantarjian H, Patel KP, Gonzalez GN, Luthra R, Kanagal Shamanna R et al. Impact of BCR-ABL transcript type on outcome in patients with chronic-phase CML treated with tyrosine kinase inhibitors. Blood 2016; 127: 1269–1275.2672989710.1182/blood-2015-10-674242PMC4786836

[bib14] Bartel DP. MicroRNAs: genomics, biogenesis, mechanism, and function. Cell 2004; 116: 281–297.1474443810.1016/s0092-8674(04)00045-5

[bib15] Calin GA, Croce CM. MicroRNA signatures in human cancers. Nat Rev Cancer 2006; 6: 857–866.1706094510.1038/nrc1997

[bib16] Kumar MS, Lu J, Mercer KL, Golub TR, Jacks T. Impaired microRNA processing enhances cellular transformation and tumorigenesis. Nat Genet 2007; 39: 673–677.1740136510.1038/ng2003

[bib17] Ventura A, Jacks T. MicroRNAs and cancer: short RNAs go a long way. Cell 2009; 136: 586–591.1923987910.1016/j.cell.2009.02.005PMC3910108

[bib18] Calin GA, Dumitru CD, Shimizu M, Bichi R, Zupo S, Noch E et al. Frequent deletions and down-regulation of micro- RNA genes miR15 and miR16 at 13q14 in chronic lymphocytic leukemia. Proc Natl Acad Sci USA 2002; 99: 15524–15529.1243402010.1073/pnas.242606799PMC137750

[bib19] Ruvkun G. Clarifications on miRNA and cancer. Science 2006; 311: 36–37.10.1126/science.311.5757.36d16400132

[bib20] Di Cristofano A, Pandolfi PP. The multiple roles of PTEN in tumor suppression. Cell 2000; 100: 387–390.1069375510.1016/s0092-8674(00)80674-1

[bib21] Stambolic V, Suzuki A, de la Pompa JL, Brothers GM, Mirtsos C, Sasaki T et al. Negative regulation of PKB/Akt-dependent cell survival by the tumor suppressor PTEN. Cell 1998; 95: 29–39.977824510.1016/s0092-8674(00)81780-8

[bib22] Li DM, Sun H. PTEN/MMAC1/TEP1 suppresses the tumorigenicity and induces G1 cell cycle arrest in human glioblastoma cells. Proc Natl Acad Sci USA 1998; 95: 15406–15411.986098110.1073/pnas.95.26.15406PMC28055

[bib23] Cha ST, Chen PS, Johansson G, Chu CY, Wang MY, Jeng YM et al. MicroRNA-519c suppresses hypoxia-inducible factor-1alpha expression and tumor angiogenesis. Cancer Res 2010; 70: 2675–2685.2023387910.1158/0008-5472.CAN-09-2448

[bib24] Iliopoulos D, Polytarchou C, Hatziapostolou M, Kottakis F, Maroulakou IG, Struhl K et al. MicroRNAs differentially regulated by Akt isoforms control EMT and stem cell renewal in cancer cells. Sci Signal 2009; 2: ra62.1982582710.1126/scisignal.2000356PMC2862216

[bib25] Zhao L, Li Y, Song X, Zhou H, Li N, Miao Y et al. Upregulation of miR-181c inhibits chemoresistance by targeting ST8SIA4 in chronic myelocytic leukemia. Oncotarget 2016; 7: 60074–60086.2752785610.18632/oncotarget.11054PMC5312369

[bib26] Testa JR, Bellacosa A. AKT plays a central role in tumorigenesis. Proc Natl Acad Sci USA 2001; 98: 10983–10985.1157295410.1073/pnas.211430998PMC58668

[bib27] Altomare DA, Wang HQ, Skele KL, De Rienzo A, Klein-Szanto AJ, Godwin AK et al. AKT and mTOR phosphorylation is frequently detected in ovarian cancer and can be targeted to disrupt ovarian tumor cell growth. Oncogene 2004; 23: 5853–5857.1520867310.1038/sj.onc.1207721

[bib28] Bockhorn J, Dalton R, Nwachukwu C, Huang S, Prat A, Yee K et al. MicroRNA-30c inhibits human breast tumour chemotherapy resistance by regulating TWF1 and IL-11. Nat Commun 2013; 4: 1393.2334043310.1038/ncomms2393PMC3723106

[bib29] Chen Y, Jacamo R, Konopleva M, Garzon R, Croce C, Andreeff M. CXCR4 downregulation of let-7a drives chemoresistance in acute myeloid leukemia. J Clin Invest 2013; 123: 2395–2407.2367650210.1172/JCI66553PMC3668829

[bib30] Vecchione A, Belletti B, Lovat F, Volinia S, Chiappetta G, Giglio S et al. A microRNA signature defines chemoresistance in ovarian cancer through modulation of angiogenesis. Proc Natl Acad Sci USA 2013; 110: 9845–9850.2369736710.1073/pnas.1305472110PMC3683704

[bib31] Yang H, Kong W, He L, Zhao JJ, O'Donnell JD, Wang J et al. MicroRNA expression profiling in human ovarian cancer: miR-214 induces cell survival and cisplatin resistance by targeting PTEN. Cancer Res 2008; 68: 425–433.1819953610.1158/0008-5472.CAN-07-2488

[bib32] Fang L, Li H, Wang L, Hu J, Jin T, Wang J et al. MicroRNA-17-5p promotes chemotherapeutic drug resistance and tumour metastasis of colorectal cancer by repressing PTEN expression. Oncotarget 2014; 5: 2974–2987.2491242210.18632/oncotarget.1614PMC4102784

[bib33] Starczynowski DT, Morin R, McPherson A, Lam J, Chari R, Wegrzyn J et al. Genome-wide identification of human microRNAs located in leukemia-associated genomic alterations. Blood 2011; 117: 595–607.2096232610.1182/blood-2010-03-277012

[bib34] Wang LS, Li L, Li L, Chu S, Shiang KD, Li M et al. MicroRNA-486 regulates normal erythropoiesis and enhances growth and modulates drug response in CML progenitors. Blood 2015; 125: 1302–1313.2551596110.1182/blood-2014-06-581926PMC4335083

[bib35] Yu Y, Yang L, Zhao M, Zhu S, Kang R, Vernon P et al. Targeting microRNA-30a-mediated autophagy enhances imatinib activity against human chronic myeloid leukemia cells. Leukemia 2012; 26: 1752–1760.2239536110.1038/leu.2012.65

[bib36] Hershkovitz-Rokah O, Modai S, Pasmanik-Chor M, Toren A, Shomron N, Raanani P et al. Restoration of miR-424 suppresses BCR-ABL activity and sensitizes CML cells to imatinib treatment. Cancer Lett 2015; 360: 245–256.2569748110.1016/j.canlet.2015.02.031

[bib37] Hershkovitz-Rokah O, Modai S, Pasmanik-Chor M, Toren A, Shomron N, Raanani P et al. MiR-30e induces apoptosis and sensitizes K562 cells to imatinib treatment via regulation of the BCR-ABL protein. Cancer Lett 2015; 356: 597–605.2530545310.1016/j.canlet.2014.10.006

[bib38] Jin G, Kim MJ, Jeon HS, Choi JE, Kim DS, Lee EB et al. PTEN mutations and relationship to EGFR, ERBB2, KRAS, and TP53 mutations in non-small cell lung cancers. Lung Cancer 2010; 69: 279–283.2001839810.1016/j.lungcan.2009.11.012

[bib39] Panigrahi AR, Pinder SE, Chan SY, Paish EC, Robertson JF, Ellis IO. The role of PTEN and its signalling pathways, including AKT, in breast cancer; an assessment of relationships with other prognostic factors and with outcome. J Pathol 2004; 204: 93–100.1530714210.1002/path.1611

[bib40] Mizoguchi M, Nutt CL, Mohapatra G, Louis DN. Genetic alterations of phosphoinositide 3-kinase subunit genes in human glioblastomas. Brain Pathol 2004; 14: 372–377.1560598410.1111/j.1750-3639.2004.tb00080.xPMC8095817

[bib41] Oda K, Stokoe D, Taketani Y, McCormick F. High frequency of coexistent mutations of PIK3CA and PTEN genes in endometrial carcinoma. Cancer Res 2005; 65: 10669–10673.1632220910.1158/0008-5472.CAN-05-2620

[bib42] Ollikainen M, Gylling A, Puputti M, Nupponen NN, Abdel-Rahman WM, Butzow R et al. Patterns of PIK3CA alterations in familial colorectal and endometrial carcinoma. Int J Cancer 2007; 121: 915–920.1747155910.1002/ijc.22768

[bib43] Mullighan CG, Goorha S, Radtke I, Miller CB, Coustan-Smith E, Dalton JD et al. Genome-wide analysis of genetic alterations in acute lymphoblastic leukaemia. Nature 2007; 446: 758–764.1734485910.1038/nature05690

[bib44] Palomero T, Sulis ML, Cortina M, Real PJ, Barnes K, Ciofani M et al. Mutational loss of PTEN induces resistance to NOTCH1 inhibition in T-cell leukemia. Nat Med 2007; 13: 1203–1210.1787388210.1038/nm1636PMC2600418

[bib45] Hollander MC, Blumenthal GM, Dennis PA. PTEN loss in the continuum of common cancers, rare syndromes and mouse models. Nat Rev Cancer 2011; 11: 289–301.2143069710.1038/nrc3037PMC6946181

[bib46] Xu J, Tang Y, Bei Y, Ding S, Che L, Yao J et al. miR-19b attenuates H2O2-induced apoptosis in rat H9C2 cardiomyocytes via targeting PTEN. Oncotarget 2016; 7: 10870–10878.2691882910.18632/oncotarget.7678PMC4905445

[bib47] Dhar S, Kumar A, Rimando AM, Zhang X, Levenson AS. Resveratrol and pterostilbene epigenetically restore PTEN expression by targeting oncomiRs of the miR-17 family in prostate cancer. Oncotarget 2015; 6: 27214–27226.2631858610.18632/oncotarget.4877PMC4694984

[bib48] Gu J, Wang D, Zhang J, Zhu Y, Li Y, Chen H et al. GFRalpha2 prompts cell growth and chemoresistance through down-regulating tumor suppressor gene PTEN via Mir-17-5p in pancreatic cancer. Cancer Lett 2016; 380: 434–441.2740068110.1016/j.canlet.2016.06.016

[bib49] Zou ZJ, Fan L, Wang L, Xu J, Zhang R, Tian T et al. miR-26a and miR-214 down-regulate expression of the PTEN gene in chronic lymphocytic leukemia, but not PTEN mutation or promoter methylation. Oncotarget 2015; 6: 1276–1285.2536101210.18632/oncotarget.2626PMC4359232

